# A Computer-Aided Method for Digestive System Abnormality Detection in WCE Images

This article has been retracted.

**DOI:** 10.1155/2021/7863113

**Published:** 2021-10-18

**Authors:** Zahra Amiri, Hamid Hassanpour, Azeddine Beghdadi

**Affiliations:** ^1^Image Processing and Data Mining Lab, Shahrood University of Technology, Shahrood, Iran; ^2^Department of Computer Science and Engineering, University Sorbonne Paris Nord, Villetaneuse, France

## Abstract

Wireless capsule endoscopy (WCE) is a powerful tool for the diagnosis of gastrointestinal diseases. The output of this tool is in video with a length of about eight hours, containing about 8000 frames. It is a difficult task for a physician to review all of the video frames. In this paper, a new abnormality detection system for WCE images is proposed. The proposed system has four main steps: (1) preprocessing, (2) region of interest (ROI) extraction, (3) feature extraction, and (4) classification. In ROI extraction, at first, distinct areas are highlighted and nondistinct areas are faded by using the joint normal distribution; then, distinct areas are extracted as an ROI segment by considering a threshold. The main idea is to extract abnormal areas in each frame. Therefore, it can be used to extract various lesions in WCE images. In the feature extraction step, three different types of features (color, texture, and shape) are employed. Finally, the features are classified using the support vector machine. The proposed system was tested on the Kvasir-Capsule dataset. The proposed system can detect multiple lesions from WCE frames with high accuracy.

## 1. Introduction

Wireless Capsule Endoscopy (WCE) is an imaging device to capture video frames from the digestive system. This technology is a noninvasive tool that has many advantages over other methods such as small-bowel imaging that is inaccessible by other traditional endoscopy methods [1]. WCE also provides realistic images from the digestive system compared with noninvasive technology such as a CT scan [2]. The captured video usually contains about 8000 frames [3].

Various lesions may appear in WCE images which are symptoms of different diseases. The most important lesions include ulcers, bleeding, lymphoid hyperplasia (LH), angiodysplasia (AD), polyps, erythematous, and erosion. Several examples of WCE frames with different lesions are shown in Figure 1. Since these lesions appear in few frames of a video and usually have a small size compared to the frame size, physicians may miss them during the examination [4]. In addition, it is a time-consuming and boring task for the physician to check a thousand frames to find pathological lesions [5]. Therefore, a computer-aided method is needed to automatically detect frames containing lesions.

In this research, a computer-aided system is proposed to detect different lesions in WCE images. Our proposed method is not limited to detecting a specific lesion and it can detect different types of lesions in WCE images. But our experiments are based on the lesions that exist in our datasets, which include bleeding (blood-fresh and blood-hematin), LH, AD, ulcers, erosion, polyps, erythematous, and foreign body.

The blood-fresh includes a red liquid that is caused by gastrointestinal (GI) bleeding. Observing small black stripes, which are due to minimal bleeding, is called blood-hematin. A rapid increase in the number of normal lymphocyte cells leads to LH. AD is a small vascular malformation of the gut. In erosion lesions, the surface of the mucosa is eroded and covered by tiny fibrin while the larger erosions are called ulcers. The tablet residue or retained capsule in the WCE images creates a foreign body class. Polyps are observable as protruding from the mucosal wall which may be precancerous lesions. Erythematous is the typical mucosal change with a reddish appearance [6].

Various challenges and limitations affect the abnormality detection system. One important issue is the high similarity among some cases in WCE frames with different lesions that complicates the detection process (see Figure 2). The quality of WCE images is lower than traditional endoscopy or colonoscopy images and also these images suffer from noise, low resolution, and blurriness [7].

As mentioned before, lesions in a frame have a small size compared to the background. It complicates the feature extraction process. Hence, it is needed to extract the small suspect region of the image as the region of interest (ROI) and then the features can be extracted from the ROI. ROI extraction is a challenging task because different lesions have various colors, shapes, and textures.

In our previous works [2, 8], the ROI extraction method was based on the expectation-maximization (EM) algorithm and it was just able to extract the red lesions from WCE frames. In this research, we propose a new method based on joint normal distribution, regardless of its color, texture, and shape, to extract distinct areas in WCE images as ROIs.

In our proposed method, we first extract ROI from the image. The main idea of the ROI extraction method is to identify distinct areas in the background by using the joint normal distribution; then, distinct areas are distinguished as the ROI segment by considering a threshold. In the next step, color, texture, and shape features are extracted from the ROI. Finally, a support vector machine (SVM) is used to classify images into different classes. In our proposed method, it is assumed that there is only one type of lesion in each WCE image. The main contributions of this study are given as follows:

- Proposing a novel method for extracting distinct regions in WCE frames as ROIs considering joint normal distribution.
- Introducing a method to classify various types of lesions in WCE images.

The rest of the paper is organized as follows: in Section 2, related works are reviewed. The proposed method is introduced in Section 3.  Section 4 discusses the experimental results. Finally, the conclusion and future works are given in Section 5.

## 2. Related Works

Several studies exist for abnormality detection in WCE images [9–15]. Most existing methods focus on identifying a specific lesion and few of them introduce a multilesion detection system for WCE images. The most common lesions in the WCE abnormality detection system are bleeding, ulcer, and AD ulcer [10–15]. According to our research, some lesions like LH and erythematous have not been investigated in any existing abnormality detection method.

Much research focused on detecting bleed in WCE frames. A bleeding detection technique in WCE images was introduced by Yuan et al. [13]. In this method, each image is described by a color histogram and it was used as a feature set for classification. The histogram was based on RGB color space but all colors were not participating in the histogram bins. Because some colors such as purple or blue are rarely seen in WCE frames, *K*-means algorithm was used to obtain the existing colors in WCE images for participating in the histogram. Caroppo et al. [14] also introduced a bleeding detection system based on deep transfer learning techniques. In this method, three popular convolutional neural network models (InceptionV3, VGG19, and ResNet50) were employed to extract features. Then, the minimum redundancy maximum relevance method was used for feature selection. Finally, the selected features were classified by supervised machine learning methods. Our proposed method is compared with these two bleeding detection methods in the result section.

Several studies exist for detecting AD lesions in WCE frames. Deeba et al. [4] introduced a saliency map-based method for AD lesion detection. The saliency map is a fusion of color and texture distinctness maps. A logarithmic ratio of the red channel to the green channel in the RGB color model creates the color map. To obtain a pattern distinctness map, the image is divided into overlapping patches and the average of all patches is calculated. Then, the distance between all patches and the average patch thorough principle axes are calculated and considered as the value of each patch in the pattern distinctness map. The accuracy of this method was considerable but this method can only be used for red lesions. In contrast, our proposed method is not limited to lesions with a specific color. Vieira et al. [15] proposed an AD detection and segmentation method based on EM based algorithm with the hidden Markov model. The Dice Score and accuracy of this method in different experiments is about 70% and 95%, respectively. The EM algorithm has an iterative manner; therefore, this method is time-consuming.

## 3. Proposed Method

In this paper, a new abnormality detection method in WCE images is proposed based on a fast ROI detection technique. The proposed system has five main steps. The steps are given below.

### 3.1. Preprocessing

There is a small boundary area in WCE images that contains some information about the capsule type and the capturing time. This area can be eliminated in the preprocessing step by applying a circular mask.

### 3.2. ROI Extraction

In each image, we need to extract distinctive regions as ROI. When the joint normal distribution model is fitted to each image, the probability of belonging each pixel in the image to the normal regions is given by a probability density function (PDF). Hence, the more probable regions can be considered as nondistinct elements and vice versa.

In this step, the ROI of each image is extracted using a fast method. For each image, the joint normal distribution of image's pixels is calculated that noted by *X* ~ *𝒩*(*μ*, Σ), *X* is three-dimensional vector *X*=[R, G, B]^*T*^ where R, G, and B are values of each image's pixels in R, G, and B components from the RGB color space, respectively. In other words, *X* is 3 × (*m*.*n*) matrix where the size of the image is (*m*.*n*). The joint normal distribution can be identified using mean vector (*μ*) and 3 × 3 covariance matrix (Σ):

(1) $$\begin{array}{c} \mu =E\left[X\right]={\left[E\left[\text{R}\right],\;E\left[\text{G}\right],\;E\left[\text{B}\right]\right]}^{T}\\ \Sigma_{i,j}=\text{Cov}\left[X_{i},X_{j}\right], \end{array}$$

where *E*[.] and Cov[., .] are expected value and covariance, respectively. Σ_*i*,*j*_ is the covariance between values of the pixels in channels *i* and *j*. Then, PDF of each image's pixel *x*=(*r*, *g*, *b*) is calculated by

(2) $$\begin{array}{c} f\left(x\right)=\frac{1}{\sqrt{{\left(2\pi \right)}^{3}\left|\Sigma \right|}}\exp\left(-\frac{1}{2}{\left(x-\mu \right)}^{T}\Sigma^{-1}\left(x-\mu \right)\right), \end{array}$$

where |.| represents the matrix determinant. The complement of *f*(*x*) can be calculated by $\bar{f\left(x\right)}=1-f\left(x\right)$.

For extracting ROI, $\bar{f\left(x\right)}$ of each pixel is calculated and pixels that have a value greater or equal to threshold *𝒯* are considered as raw ROI.

Our results show that the raw ROI segment has small blobs or lines; hence, these areas must be removed. To remove these areas, we firstly used an opening morphology filter with a disk structuring element of radius six. Eccentricity shows the dissimilarity between a blob and a circle [16]. If the eccentricity is near to zero, the blob is similar to a circle and when it is near to one, the blob is similar to a line. Lesions are dissimilar to the line; therefore, the blobs smaller than 100 pixels or eccentricity >0.9 will be removed from the raw ROI segment.

### 3.3. Feature Extraction

In this step, three types of features including color, shape, and texture are extracted. The color features are extracted from each component of RGB, HSV, and LAB color modes. In each component, eight different features including mean, minimum, maximum, variance, mode, entropy, median, and contrast are extracted from ROI. Therefore, 9 × 8=72 color features are extracted in this part.

For extracting shape features, a histogram of oriented gradients (HOG) is used. In this part, the lowest possible rectangle that contains the whole ROI is selected. Then, this area is resized to 48 × 48. Finally, the HOG of this resized area is calculated. The parameters of HOG are given in Table 1. Based on these parameters, there are 6 × 6=36 patches. Therefore, 36 × 5=180 shape features are extracted in this part.

LBP is one of the famous methods for extracting texture features [17, 18]. The uniform LBP [19] is a rotation-invariant version of LBP. In the last part, uniform LBP is calculated as texture features from ROI (non-ROI regions are set to zero). This feature was used in many WCE classification methods [20, 21]. We used uniform LBP with 3 × 3 neighboring blocks. Comparing each pixel with its neighbors generates an 8-digit binary number. Therefore, 256 different numbers can be created. In the LBP method, the histogram of these numbers is calculated as a feature vector. In the uniform LBP, these 256 numbers are divided into uniform (they have at most two 0-1 or 1-0 transitions in an 8-digit binary number) and nonuniform patterns. Each uniform pattern has a separated bin in the final histogram, but only a single bin is assigned to nonuniform patterns. So, the feature vector length is reduced to 59 in uniform LBP.

### 3.4. Feature Selection

In this step, the correlation-based feature selection (CFS) methodology is used for finding relevant features [22], which is a well-known method. In the CFS method, some subsets of features are evaluated based on one hypothesis that the features in good feature subsets are highly correlated with the classification, but they are not uncorrelated to each other. In our method, the subset of features is searched using the greedy hill-climbing and backtracking method [23]. The search is started with an empty subset and forward direction.

### 3.5. Classification

In this step, the extracted features are classified using SVM [24, 25]. In the SVM method, a polynomial kernel with degree two is used. For more generality, *k*-fold cross-validation [26] is used for reporting results. In k-fold cross-validation, the images are divided into *k* groups. The model is trained *k* times. In each iteration, one group is separated for validation and the remaining are used for training. In each training phase, the evaluation criteria are calculated on the validation set. Each group is considered as the validation only once. Finally, the average of all calculated evaluation criteria is considered by k-fold cross-validation.

## 4. Results and Discussion

In this section, the proposed method is implemented and applied on three datasets; then, experimental results are given.

### 4.1. Dataset

We evaluate and compare our proposed method in three different datasets including the Kvasir-Capsule [6], red lesion endoscopy dataset [27], and gastrointestinal image analysis challenge 2017 [28].

Kvasir-Capsule is a publicly released WCE dataset with different labeled images; it was created in 2020 and updated in 2021 [6]. The Kvasir-Capsule dataset is split into three: (I) labeled image data, (II) labeled video data, and (III) unlabeled video data parts. In this paper, we used labeled image data. In this part, there are 47,238 images from different classes. The details are listed in Table 2. Among these classes, the ileocecal valve, pylorus, and ampulla of Vater are in the anatomy category and the reduced mucosal view contains frames that the view of the mucosa is reduced because of some existing contents like stool or bubbles. The rest of the classes belongs to normal and different pathological findings (angiectasia, erosion, ulcer, polyp, hematin, foreign bodies, erythematous, and blood). Some examples of dataset images are given in Figure 3. We applied the proposed method to the normal class and the other pathological findings classes showing the ability of the proposed method in abnormality detection in WCE images. Additionally, for balancing the dataset, we used only 1000 normal images randomly. The size of WCE frames in this dataset is 336 × 336 pixels.

The second database consists of 3895 images in 320 × 320 pixels, containing 2325 normal and 1570 bleeding frames. One binary ground truth mask exists for each frame. Two samples of this dataset images are shown in Figure 4. The third dataset consists of 600 normal and 600 abnormal images with AD lesions. One binary ground truth mask exists for each image as shown in Figure 5. The size of these images is 704 × 704 pixels.

### 4.2. Experimental Results

In the first step, all images are resized to 320 × 320 pixels and then a binary mask is applied to the images for eliminating the border area around the image. This mask is shown in Figure 6. In some datasets for the privacy of patients, this information was removed by the publisher. However, this step is proposed by the authors because of the generality of the proposed system.

In the second step, the joint normal distribution of each image is calculated. The PDF of two sample images is shown in Figure 7(b). Complement of *f*(*x*) and the raw ROI are given in Figures 7(c) and 7(d). Finally, the extracted ROIs are given in Figure 7(e). As can be seen, the extracted ROI contains the lesion position with some additional areas. In the third step, 310 features from ROI are extracted. Finally, the features are given to SVM to classify the image into different classes. We used a 10-fold cross-validation algorithm for the generalization of the results. In this paper, accuracy, false negative rate (FN rate or miss rate), false positive rate (FP rate), precision, recall, *F*-measure Dice Score (DS), and Intersection over Union (IoU) are used for evaluation of the results. The formula of these metrics is listed as follows:

(3) $$\begin{array}{c} \mathrm{AC=}\frac{\mathrm{TP+TN}}{\mathrm{TP+TN+FP+FN}}, \end{array}$$

(4) $$\begin{array}{c} \mathrm{FPR=}\frac{\mathrm{FP}}{\mathrm{FP+TN}}, \end{array}$$

(5) $$\begin{array}{c} \mathrm{FPR=}\frac{\mathrm{FP}}{\mathrm{FP+TN}}, \end{array}$$

(6) $$\begin{array}{c} \mathrm{Precision=}\frac{\mathrm{TP}}{\mathrm{TP+FP}}, \end{array}$$

(7) $$\begin{array}{c} \mathrm{Recall=Sensivisity=}\frac{\mathrm{TP}}{\mathrm{TP+FN}}\mathrm{=1-FNR,} \end{array}$$

(8) $$\begin{array}{c} F\mathrm{-Measure=2}\frac{\mathrm{Precision*Recall}}{\mathrm{Precision+Recall}}, \end{array}$$

(9) $$\begin{array}{c} \mathrm{DS=}\frac{\mathrm{2TP}}{\mathrm{2TP+FP+FN}}, \end{array}$$

(10) $$\begin{array}{c} \mathrm{IoU=}\frac{\mathrm{TP}}{\mathrm{TP+FP+FN}}, \end{array}$$

In these equations, TP, FP, TN, and FN are true positive, false positive, true negative, and false negative, respectively.

To continue, firstly, we evaluated our ROI extraction method in terms of DS and IoU and compared it with other deep learning methods. Then, our proposed abnormalities detection system was evaluated on the Kvasir dataset with different evaluation metrics. In the next experiment, the time complexity of the method was evaluated. Then, the effectiveness of different steps in the proposed method was tested. We also designed an experiment to investigate the relationship between lesions size and accuracy of the method. Finally, our proposed method was compared with four other methods on the second and third datasets.

ROI extraction is an important step in our proposed abnormality detection method that affects the final classification accuracy. Therefore, we evaluated our ROI extraction method in terms of DS and IOU in the third dataset and reported them in Table 3. References [29, 30] also used deep learning methods to segment AD lesions. These methods were evaluated in terms of DS and IoU on the third dataset. So, we also showed the results of these two methods in Table 3 to compare them with our proposed method. The results in this table showed that our proposed method had a better performance in terms of DS and IoU.

To evaluate our abnormalities detection method, our proposed method was tested on the Kvasir dataset. The results are given in Table 4 and the corresponding confusion matrix is reported in Table 5. The results showed the proposed method was able to detect different abnormalities in WCE with high accuracy. It was notable that the number of features selected by the feature selection algorithm was 64. The selected feature set were 36 from color, 5 from shape, and 23 from texture.

In this paper, a fast digestive system abnormalities detection method was proposed. To estimate the computational complexity, the proposed method was applied 1000 times on each image and the average running time was calculated. Our experiments were performed on a personal computer (see Table 6). The average processing time was 0.071 seconds. This short time shows that the proposed method was fast enough to be considered a real-time method.

In the next experiment, we investigated the effectiveness of different steps of the proposed method containing the ROI extraction step, feature extraction step, and feature selection step. To prove the positive impact of the ROI extraction step, the features were extracted from the whole part of the images. The results reported in the second row of Table 7 showed that the elimination of this step had led to a decrease in all evaluation criteria. It is notable that, in Table 7, we reported the weighted average of the metric in all ten existing classes of the first dataset. In the next investigation, we removed the feature selection step, and the results are reported in the third row of Table 7. The results showed that feature selection not only reduced the number of features but also increased the performance of the method. Finally, the effect of removing each feature type was evaluated. From the results in the fourth to the sixth rows of Table 7, it can be concluded that all types of features had a positive effect on the performance of the method, but the color feature had the most effect and the shape effect has the least effect.

In the next experiment, the impact of lesions size on the performance of the method was investigated. In this experiment, for each class in the first dataset, the average size of lesions with respect to the frame size was calculated. These averages values for different classes from smallest to the largest lesion were sorted and then the value of *F*-measure for these classes was calculated as reported in Figure 8. As can be deducted from Figure 8, there was no relation between the lesion size and method performance in our proposed method.

The proposed method was compared with our previous work in [2] and Yuan's method [13]. The methods were applied to the third dataset and the results are reported in Table 8. As can be seen, the proposed method outperformed the other two methods in all evaluation criteria and the results of Yuan's method were not acceptable on this dataset but our previous work had better results than Yuan's method.

In addition, the proposed method was compared with a deep transfer learning method [14]. The authors reported their results on the second dataset. Therefore, the proposed method is also applied to this dataset and the results are reported in Table 9. As can be seen, the proposed method shows better performance based on all metrics.

Finally, we compared the proposed method with Deeba et al.'s method [4] in all introduced evaluation metrics on the second and third datasets. It should be noted that the implementation code of this method was shared in GitHub (https://github.com/Farah-Deeba/Angiectasia-Detection) by the authors. As can be seen from Table 10, the proposed method had performed better in all evaluation criteria.

## 5. Conclusion

In this paper, a new method was proposed for abnormality detection in WCE images. The proposed method is based on four main steps: preprocessing, ROI extraction, feature extraction, and classification. In this paper, a fast ROI extraction based on joint normal distribution is proposed. The ROI extraction method distinguishes the suspect region from the background for possible abnormality detection. The proposed method was tested on three different datasets. The results show the ability of the proposed method on abnormalities detection in WCE images. Also, the proposed method is compared with several existing methods for lesion detection, and in all comparisons, the superiority of the proposed method is concluded.

## Figures and Tables

**Figure 1:** Sample WCE images: from left to right and top to bottom: normal frame, frame with AD, LH, ulcer, bleeding, polyp, erosion, and erythematous lesion. The lesion area is specified in a red circle.

**Figure 2:** High similarity among WCE images in different classes. The AD lesion is marked in a circle.

**Figure 3:** Some examples of Kvasir dataset images: (a) angiectasia, (b) erosion, (c) lymphoid hyperplasia, (d) ulcer, (e) polyp, (f) blood-hematin, (g) foreign bodies, (h) erythematous, (i) blood-fresh, and (j) normal frame. In each part, the left image is the WCE image and the right image is the corresponding mask.

**Figure 4:** Some examples of red lesion endoscopy dataset images: (a) bleeding and (b) normal.

**Figure 5:** Some examples of gastrointestinal image analysis challenge 2017 images: (a) angiectasia and (b) normal.

**Figure 6:** The applied mask.

**Figure 7:** ROI extraction step on two different WCE images. The rows are from top to button an image with LH lesion and an image with AD lesion: (a) WCE image, (b) PDF of image's pixel (*f*(*x*)), (c)$\bar{f\left(x\right)}=1-f\left(x\right)$, (d) raw extracted ROI, (e) extracted ROI, (f) correct lesion position.

**Figure 8:** Relation between lesion size and *F*-measure.

**Table 1:** Parameters of HOG.

Parameter	Value
Cell size	8 × 8
Number of bins	5
Overlapping	Nonoverlap

**Table 2:** Kvasir-Capsule dataset.

Class	Number of images
Angiectasia	866
Ampulla of Vater	10
Erosion	506
Lymphoid hyperplasia	592
Ulcer	854
Reduced mucosal view	2906
Pylorus	1529
Polyp	55
Ileocecal valve	4189
Hematin	12
Foreign bodies	776
Erythematous	139
Blood	446
Normal mucosa	34,338

**Table 3:** Comparison of the proposed method, Gobpradit's method [30], and Shvets's method [29].

Method	Shvets's method [29]	Gobpradit's method [30]	Proposed method
DS	84.98	86.17	86.87
IoU	75.35	76.64	76.79

**Table 4:** The results of classification on Kvasir dataset.

Class ↓ /metric ⟶	Accuracy	FN rate	FP rate	Precision	Recall	*F*-measure
Angiectasia	0.973	0.066	0.019	0.906	0.934	0.920
Blood-fresh	0.992	0.034	0.005	0.945	0.966	0.956
Hematin	0.999	0.167	0.000	1.000	0.833	0.909
Erosion	0.951	0.273	0.025	0.759	0.727	0.743
Erythematous	0.989	0.232	0.005	0.797	0.768	0.782
Foreign bodies	0.999	0.004	0.001	0.994	0.996	0.995
Lymphoid hyperplasia	0.981	0.081	0.011	0.916	0.919	0.917
Polyp	0.999	0.091	0.001	0.943	0.909	0.926
Ulcer	0.973	0.090	0.015	0.921	0.910	0.915
Normal mucosa	0.934	0.169	0.040	0.832	0.831	0.831

**Table 5:** Confusion matrix.

Class ↓ /classified as ⟶	C1	C2	C3	C4	C5	C6	C7	C8	C9	C10
Angiectasia (C1)	809	10	0	18	0	0	3	2	5	19
Blood-fresh (C2)	13	431	0	0	0	0	1	0	1	0
Hematin (C3)	0	0	10	0	0	2	0	0	0	0
Erosion (C4)	21	7	0	368	4	0	6	0	23	77
Erythematous (C5)	4	0	0	7	106	0	0	0	4	17
Foreign bodies (C6)	0	0	0	0	0	773	1	0	0	2
Lymphoid hyperplasia (C7)	5	0	0	11	2	0	544	0	1	29
Polyp (C8)	1	0	0	0	0	0	1	50	0	3
Ulcer (C9)	17	5	0	24	7	0	3	0	777	21
Normal mucosa (C10)	23	3	0	57	14	3	35	1	33	831

**Table 6:** The properties of the experimental setup.

Parameter	Description
CPU	Intel (R) Core (TM) i5-6100U CPU @ 2.30 GHz
RAM	8 GB
Operating system	Microsoft Windows 10
Compiler	MATLAB 2016

**Table 7:** The effectiveness of different steps of the proposed method.

Method ↓ /metric ⟶	Accuracy	TN rate	FP rate	Precision	Recall	*F*-measure
Proposed method	0.896	0.1049	0.018	0.895	0.896	0.895
Remove ROI extraction	0.832	0.1680	0.030	0.830	0.832	0.830
Remove feature selection	0.878	0.1220	0.020	0.879	0.878	0.877
Remove color features	0.707	0.293	0.054	0.713	0.707	0.705
Remove texture features	0.822	0.1780	0.032	0.818	0.822	0.817
Remove shape features	0.878	0.1220	0.021	0.877	0.878	0.877

**Table 8:** Comparison of the proposed method, Yuan's method [13], and our previous work [2].

Method ↓ /metric ⟶	Accuracy	FNR	FPR	Precision	Recall	*F*-measure
Proposed method	0.954	0.048	0.043	0.956	0.952	0.954
Yuan's method [13]	0.690	0.226	0.477	0.765	0.774	0.769
Our previous method [2]	0.895	0.099	0.115	0.940	0.901	0.920

**Table 9:** Comparison of the proposed method and Caroppo et al.'s method [14].

Method ↓ /metric ⟶	Accuracy	FNR	FPR	Precision	Recall	*F*-measure
Our proposed method	0.984	0.009	0.033	0.985	0.991	0.988
Caroppo et al. [14]	0.957	0.042	0.047	0.970	0.958	0.964

**Table 10:** Comparison of the proposed method and Deeba et al.'s method [4].

Dataset	Third dataset	
Metric ↓ /method ⟶	Deeba et al.'s method [4]	Proposed method
Accuracy	0.667	0.954
Recall	0.554	0.952
FNR	0.446	0.048
FPR	0.314	0.043
DS	52.4	86.87
IoU	41.35	76.79
Test time (seconds)	1.24	0.071

## Data Availability

The first dataset analyzed during the current study is available in the Kvasir-Capsule dataset repository (https://osf.io/dv2ag/). The second dataset analyzed during the current study is available in the red lesion endoscopy dataset (https://rdm.inesctec.pt/dataset/nis-2018-003). The third dataset analyzed during the current study is available in the GIANA challenge (https://endovissub2017-giana.grand-challenge.org/).
